# The Use of Medium‐Deep Peelings to Treat Melasma: A Case Series Study

**DOI:** 10.1111/jocd.70291

**Published:** 2025-08-18

**Authors:** Maria Tereza Scardua, Natália Scardua, Maria Fernanda Ismail, Wilson Bambirra Junior, Inês Maria Candeias Carpinteiro, Andréia Luiza Oliveira Costa, André Luiz Sena Guimarães

**Affiliations:** ^1^ Tereza Scardua Institute São Paulo São Paulo Brazil; ^2^ Department of Dentistry Universidade Estadual de Montes Claros (Unimontes) Montes Claros Minas Gerais Brazil; ^3^ Egas Moniz Center for Interdisciplinary, Research (CiiEM) Egas Moniz School of Health & Science Portugal

**Keywords:** facial melasma, heatmap visualization techniques, melasma treatment outcomes, peels, pigmentation, quantitative image evaluation, retrospective cohort study, segmented chemical peels, skin pigmentation analysis

## Abstract

**Objective:**

To evaluate the efficacy and safety of medium‐deep chemical peels for melasma in a diverse population using quantitative and subjective methodologies for comprehensive outcome assessment.

**Methods:**

A case series of 42 melasma region treatments was conducted from March 2023 to December 2024. Treatments included 30% phenol with 0.8% croton oil or a two‐step protocol of 30% glycolic acid followed by 35% trichloroacetic acid (TCA) with 0.7% croton oil. Quantitative pigmentation analysis utilized the weighted skin intensity (WSI) ratio via Fiji ImageJ software. A panel of 20 experts conducted subjective evaluations based on standardized photographs, rating pigmentation reduction, skin tone uniformity, and overall appearance. Statistical analyses included the Wilcoxon signed‐rank test and heatmap visualizations.

**Results:**

Quantitative analysis showed significant improvements in pigmentation, with mean WSI values increasing from 78.99 ± 19.58 (untreated) to 88.33 ± 22.05 (treated; *Z* = −5.495), *p* < 0.001). Heatmaps confirmed uniform pigmentation reductions. Among 42 treatments, 38 showed positive changes (*Z* = −5.092, *p* < 0.001). Experts identified 94.4% of cases as post‐treatment and rated pigmentation reduction as Grade 4 or 5 in 87.5% of responses, with similarly high ratings for skin tone uniformity (69.4%) and overall appearance (79.4%).

**Conclusion:**

Medium‐to‐deep chemical peels, utilizing phenol‐croton oil or TCA, demonstrated significant efficacy in reducing pigmentation, enhancing skin regeneration, and improving overall skin quality. Quantitative analysis and specialized clinical assessments confirmed their role as a targeted and effective approach for melasma treatment. These findings support using medium‐to‐deep peels as a personalized therapeutic strategy, offering a scientifically validated option for managing refractory melasma.

## 1 Introduction

Melasma is a common, chronic hyperpigmentation disorder that predominantly affects sun‐exposed areas, especially the face [1, 2]. It is more prevalent in women of reproductive age with Fitzpatrick skin types III–V and has a significant psychosocial impact due to its effect on facial appearance [3]. The condition affects 15%–35% of adult women in regions with high ultraviolet (UV) exposure, such as intertropical areas, with genetic predisposition and environmental triggers playing critical roles in its pathogenesis [2, 4]. Melasma is a multifactorial condition driven by environmental, hormonal, genetic, and cellular factors, leading to persistent hyperpigmentation [5, 6, 7, 8]. Beyond increased melanocyte activity, its pathogenesis involves keratinocytes, senescent fibroblasts, mast cells, endothelial cells, and basement membrane disruption [5, 6, 7, 8]. UV radiation remains a key trigger, activating pathways like protein kinase A (PKA) and microphthalmia‐associated transcription factor (MITF) to increase melanin production [5, 6, 7, 8]. Crucially, basement membrane degradation by matrix metalloproteinases (MMPs) allows melanocytes to migrate into the dermis, making melasma more resistant to treatment [5, 6, 7, 8]. Effective management should target pigment reduction and restore basement membrane integrity to prevent melanocyte infiltration, reduce inflammation, and enhance treatment outcomes [5, 6, 7, 8]. UV radiation is the most significant external trigger, intensifying melanogenesis through increased cytokine production and stem cell factor signaling [2, 9]. Hormonal influences, particularly elevated estrogen and progesterone levels during pregnancy or oral contraceptive use, are also strongly implicated in its onset and persistence [10]. Furthermore, genetic factors, including family history and specific gene expressions like TYRP1 and Wnt pathway modulators, underscore the hereditary aspect of melasma [11].

Histologically, melasma is characterized by increased melanin deposition in the epidermis and dermis, basal membrane disruption, and extracellular matrix (ECM) changes, including solar elastosis [5, 12]. Recent studies highlight the role of oxidative stress, vascular alterations, and neuropeptide activity in the pathophysiology, suggesting that melasma is not merely a pigmentary disorder but a manifestation of dermal and epidermal dysfunction [5].

Chemical peels, including phenol‐croton [13], glycolic acid, salicylic acid, and trichloroacetic acid (TCA) [14], are widely utilized as second‐line treatments to address the epidermal component of melasma. These agents induce controlled exfoliation and promote epidermal remodeling, removing melanin‐laden keratinocytes and dermal reorganization. Recent studies suggest combining chemical peels with other modalities, such as topical depigmenting agents and rigorous photoprotection, yield better therapeutic outcomes by targeting multiple pathways involved in melasma pathogenesis [13, 14]. Medium‐to‐deep chemical peels offer a promising approach for melasma treatment by targeting both the epidermis and dermis [5, 6, 7, 8]. These peels work through a dual mechanism: removing pigmented keratinocytes while promoting profound tissue remodeling [5, 6, 7, 8]. Reaching the upper reticular dermis stimulates neocollagenesis and elastogenesis, eliminates senescent cells, and reverses solar elastosis [5, 6, 7, 8]. Crucially, they help restore the basement membrane, preventing melanocyte migration into the dermis and reducing chronic inflammation [5, 6, 7, 8]. This profound restructuring of the ECM balances melanogenesis and enhances skin regeneration, providing a long‐lasting and effective treatment for severe melasma and advanced photoaging [5, 6, 7, 8].

These peels target epidermal and dermal components, reducing pigmentation and improving skin structure. This case series comprehensively evaluates medium‐deep chemical peels in refractory melasma by combining objective image analysis with expert assessments.

## 2 Methods

### 2.1 Study Design and Setting

This retrospective case series study was conducted at a reference center. The study included patients diagnosed with melasma who underwent segmented chemical peel treatments between March 2023 and December 2024. The institutional ethics committee approved the study protocol 82464024.9.0000.5146, and all procedures adhered to the principles of the Declaration of Helsinki. The study was reported according to Preferred Reporting of Case Series in Surgery (PROCESS) guidelines [15] (Supporting Information S1).

### 2.2 Segmented Chemical Peeling Protocol

The chemical peeling procedures were performed by two trained clinicians using a segmented approach. Segmented chemical peeling refers to applying the peel to specific facial areas at different times. This strategy was selected to enhance safety and provide better control during healing. Limiting medium‐to‐deep peel application to smaller areas made the postoperative period more manageable and less aggressive for the patient, allowing for closer and more effective clinical monitoring. Furthermore, this segmentation facilitated the management of potential complications—such as bacterial infections, herpes simplex outbreaks, or fungal overgrowth—by reducing the treated surface area and improving the clinician's ability to detect and respond to adverse events during recovery. The facial areas treated in a segmented manner included:

Forehead: Treatment extended up to the mid‐temporal regions, irrespective of the extent of hyperpigmentation.

Malar regions: The entire malar (cheek) area was treated, from the lower eyelid margin to the inferior mandibular border.

Upper lip and perioral region: Treatment encompassed the area from the nasal base to the inferior mandibular margin, extending approximately 1 cm beyond the oral commissures.

By restricting the extent of skin subjected to medium‐ to deep‐depth chemical peels at each session, the segmented approach allowed for more precise postoperative monitoring. It facilitated early identification and management of potential complications, such as bacterial, herpetic, or fungal infections. The control of the treated area consequently reduced risks during the healing process. Following the initial recovery period, clinical evaluations assessed the degree of reduction in hyperpigmentation and erythema. Additional segmented peel sessions were performed following the same protocol to optimize aesthetic outcomes when necessary. In some instances, residual pigmentation remained due to the depth of melasma or the layer reached by the peeling agent; one to two additional sessions were sometimes required to achieve more uniform results. In some patients, the untreated areas of the face were subsequently addressed to harmonize color and texture, particularly when noticeable contrast was observed between treated and untreated skin. The decision to treat additional regions was based on the degree of skin aging and tanning intensity rather than solely on the phototype. This individualized approach ensured more balanced and esthetically pleasing results.

### 2.3 Ingredients and Preparation of Peeling Solutions

The peeling solutions were prepared by the compounding pharmacy, considering each patient's skin thickness and specific needs. Two distinct formulations were employed to ensure optimal treatment efficacy. The first formulation consisted of 30% phenol and 0.8% croton oil. The second formulation followed a two‐step protocol, beginning with applying 30% glycolic acid, followed by a mixture of TCA at either 35% or 0.7% croton oil. These customized solutions were specifically designed to tailor the peeling depth and intensity according to the individual characteristics of each patient's skin, thereby enhancing both safety and clinical outcomes.

### 2.4 Postoperative Care and Healing

Immediately following the chemical peeling procedure, a protective chemical mask containing 1% lidocaine, 100 000 IU/g nystatin, and a plastic barrier layer was applied over the treated areas. This mask was maintained for 3 days to protect the skin and facilitate the initial stages of healing. Patients were instructed to gently remove the mask by softening it with water during bathing, thereby minimizing mechanical trauma to the newly treated skin. During the subsequent healing phase, patients were advised to apply a topical collagenase ointment combined with chloramphenicol twice daily and petroleum jelly (vaseline) to maintain adequate skin hydration and support the regenerative process.

### 2.5 Microneedling and Management of Post‐Inflammatory Hyperpigmentation

Microneedling was systematically performed in all patients who developed post‐inflammatory hyperpigmentation (PIH) between 15 and 30 days following the chemical peeling procedure. The microneedling protocol consisted of two stages. In the first stage, microneedling was performed in conjunction with the application of 0.3–0.5 mL of hyaluronidase (500 units diluted in 3 mL of physiological saline solution), aiming to disrupt the ECM and thereby enhance the penetration and efficacy of subsequently applied active agents [16]. Immediately following microneedling, a specially formulated topical solution was used, composed of 10% hydroquinone, 2% salicylic acid, 10% resorcinol, 5% phytic acid, 1% D‐panthenol, and a 30% blend of alpha hydroxy acids. The integration of segmented chemical peeling with targeted microneedling thus provided an effective and customizable therapeutic strategy for treating PIH.

### 2.6 Sample Population

The study analyzed 42 sites of melasma across diverse skin phototypes. Of a total of participants, 35 patients were treated exclusively with phenol/croton oil peels, two patients received glycolic acid/TCA/croton oil peels, and seven patients began with phenol/croton oil peels and later transitioned to glycolic acid/TCA/croton oil peels. Participants were required to have a confirmed clinical diagnosis of melasma and complete treatment records with follow‐up data. All patients underwent segmented chemical peels as part of their treatment regimen and were monitored over an average follow‐up period of 256 days, ensuring a comprehensive evaluation of treatment outcomes.

### 2.7 Inclusion and Exclusion Criteria

Patients with a clinically confirmed diagnosis of melasma affecting any facial area regardless of skin phototype or age, who had previously undergone unsuccessful treatment attempts, were included in the study. Exclusion criteria comprised the presence of active infections in the treatment area, a history of severe adverse reactions to chemical peels, the use of immunosuppressive medications, pregnancy or lactation, active autoimmune diseases, or refusal to sign the informed consent form.

### 2.8 Outcome Measures

The photos were taken using a digital single‐lens reflex (DSLR) camera (Canon EOS 80D, Canon Inc., Tokyo, Japan) with a 50 mm lens under consistent lighting. The camera settings were as follows: ISO 2500, shutter speed 1/60, and aperture f/7.1. The autofocus operation was set to “One Shot,” and the images were saved as JPEG files with a resolution of 6000 × 4000 pixels. The white balance was configured at B4, G5/+0, and the picture style was set to “Auto” to ensure standardized image quality across all captures. To enable accurate comparisons, a small area of untreated skin was systematically preserved in each patient until the final assessment, serving as a standardized internal control for baseline skin color and texture. Changes in melasma pigmentation were quantified using Fiji ImageJ software [17], a validated tool for image analysis [18, 19]. The study focused on the weighted skin intensity (WSI) ratio, a quantitative measure of variations in skin tone or color intensity. This ratio is calculated by assigning specific weighted values to intensity parameters such as brightness, hue, and saturation within the sampled skin area. Results are expressed as percentages, representing the relative contribution of each intensity level to the overall skin profile. This approach provides a reliable framework for evaluating and comparing skin conditions or treatment effects.

The WSI ratio was computed using Fiji's Histogram function, which analyzes intensity levels ranging from 0 to 255. Higher values correspond to tones closer to white, while lower values represent darker tones. High‐resolution photographs were taken using DSLR cameras under standardized lighting and environmental conditions to ensure consistency.

For each analyzed region, two measurements were performed: one for the lesion or treated area and one for a control region unaffected by melasma. The percentage of intensity weighted for the lesion or treated area was calculated relative to the control region (Figure 1). Additionally, a heatmap was created to visualize changes by calculating the total percentage of intensity weighted as the ratio of post‐treatment to pre‐treatment measurements. This process provided an objective and detailed evaluation of the treatment's effectiveness in modifying skin pigmentation and texture (Figure 1).

**FIGURE 1:** Weighted skin intensity (WSI) calculation scheme. Schematic illustration of the image analysis protocol for quantifying pigmentation changes. In the pre‐treatment image (left panel), region (A) corresponds to the melasma‐affected area, and region (B) corresponds to the untreated control area. In the post‐treatment image (right panel), region (C) corresponds to the area subjected to treatment, while region (D) corresponds to the untreated area preserved as a post‐treatment control. Quantitative comparisons were performed by calculating intensity ratios between treated and untreated regions at both time points.

A panel of experts conducted subjective analyses. Using the online software Research Randomizer (Version 4.0) (https://www.randomizer.org), eight regions were randomly selected from 42 areas. A questionnaire was then distributed via Google Forms to the experts for their assessment. Each case was presented as an image without captions, and the experts were asked to determine which side they believed represented the post‐treatment condition (options: right or left). Additionally, they rated various aspects of the treatment outcomes on a scale of 1–5, where higher scores indicated better results. These aspects included the visible reduction in melasma pigmentation, skin tone uniformity, reduction of visible borders of melasma patches, overall skin appearance (texture and luminosity), and a global evaluation of the treatment results. The experts were blinded to all clinical details, including the type of treatment performed, the time between sessions, and any other procedural information, analyzing only before‐and‐after photographs, which had been aligned and standardized using artificial intelligence to prevent any manipulation of the images. The selected cases were thoroughly assessed by 20 experts, providing valuable insights into the treatment's effectiveness across multiple qualitative and quantitative dimensions. We analyzed every session separately to evaluate the results of each treatment. Melasma severity was measured using the Modified Melasma Area and Severity Index (MASI), a standard tool for assessing melasma. We used high‐quality photographs taken just before each treatment to apply this scoring system [20].

### 2.9 Statistical Analysis

The Shapiro–Wilk and Kolmogorov–Smirnov tests were conducted to assess the normality of data distribution. Since the data did not follow the parametric distribution and the measurements were related, the Wilcoxon signed‐rank test was applied for statistical analysis using Statistical Package for the Social Sciences (SPSS) software (IBM SPSS Statistics for Windows, Version 22.0. Armonk, NY, USA). A heat map was generated to compare the pre‐treatment, post‐treatment, and total percentage of intensity‐weighted values, utilizing GraphPad Prism (version 8.0.1 for Windows, GraphPad Software, Boston, Massachusetts, USA). Statistical significance was defined as (*p* < 0.05).

## 3 Results

### 3.1 Demographic Data

The study analyzed 42 facial melasma sites from 35 female patients aged between 36 and 74 (mean age: 48.8 years). While ethnicity was not explicitly recorded, the Fitzpatrick skin phototype distribution—used as an indicator of skin response to UV radiation—showed a predominance of phototypes IV (*n* = 18, 42.9%) and III (*n* = 17, 40.5%), followed by phototype V (*n* = 4, 9.5%) and phototype II (*n* = 3, 7.1%). The mean MASI score at baseline was 3.90. Most cases were classified as mild (*n* = 32, 76.2%), with moderate (*n* = 6, 14.3%) and severe (*n* = 4, 9.5%) cases being less frequent (Supporting Information S2). It is essential to highlight that although 35 patients were enrolled, multiple facial sites were assessed for WSI analysis, allowing for the evaluation of 42 distinct melasma presentations across various skin phototypes.

### 3.2 Changes in WSI Ratio

The efficacy of medium‐deep chemical peels for treating melasma was evaluated quantitatively using Fiji ImageJ software, focusing on the WSI ratio (Figure 2). The analysis demonstrated significant improvements in treated areas compared to untreated regions. Descriptive statistics revealed that untreated areas had a mean intensity value of 78.99 ± 19.58. In contrast, treated areas showed a higher mean intensity value of 88.33 ± 22.05, indicating a shift toward lighter skin tones post‐treatment (higher WSI values). The Wilcoxon signed‐rank test compared intensity values before and after treatment, revealing a statistically significant improvement in treated areas (*Z* = −5.495, *p* < 0.001); Figure 2A). Among the 42 cases analyzed, 38 exhibited positive changes in skin tone (Figure 2B), while four cases showed negative changes, with no ties observed. The Sign Test corroborated these findings, confirming a significant difference between treated and untreated regions (*Z* = −5.092, *p* < 0.001). Overall, 38 of the 42 cases showed improvements, highlighting the treatment's effectiveness. The Marginal Homogeneity Test further supported these results, showing significant consistency in the observed improvements across cases (*p* < 0.001, data not shown). Heatmaps generated from the intensity‐weighted data visually represented pigmentation changes, with treated areas demonstrating uniform reductions in pigmentation. The heatmaps, particularly in regions with higher baseline melasma intensity, emphasized the transition toward lighter colors, consistent with improved skin tone (Figure 2B). These findings from both quantitative and visual analyses underscore the significant impact of medium‐deep chemical peels in reducing melasma pigmentation and enhancing skin tone and texture.

**FIGURE 2:** Quantitative evaluation of the efficacy of medium‐deep chemical peels for melasma treatment. In (A) presents a comparison of weighted skin intensity (WSI) ratios between treated and untreated areas, demonstrating a significant increase in WSI values post‐treatment (Wilcoxon signed‐rank test, *Z* = −5.495, *p* < 0.001). Untreated areas exhibited a mean WSI of 78.99 ± 19.58, whereas treated areas showed a higher mean WSI of 88.33 ± 22.05, indicating lighter skin tones. (B) Heatmap representation of WSI percentages, illustrating the intensity‐weighted pigmentation changes at three‐time points: Pre‐treatment (PR), after treatment (AR), and the treatment ratio (TR). The heatmaps highlight uniform reductions in pigmentation and confirm the effectiveness of the treatment across cases.

### 3.3 Subjective Analysis

A panel of 20 experts conducted a subjective evaluation of medium‐deep chemical peels for melasma treatment using standardized in Figure 3, anonymized before‐and‐after images from eight randomly selected cases. The experts, blinded to all procedural details, assessed various aspects of the treatment outcomes, providing overwhelmingly positive feedback. They correctly identified the post‐treatment condition in 94.4% of cases (Figure 3A), reflecting the visible improvements achieved. 87.5% of responses were rated as Grade 4 or 5 for the reduction in melasma pigmentation, indicating significant improvement, with 50% rated as Grade 5 (Figure 3B). Similarly, 69.4% of responses for skin tone uniformity were rated in the top two categories, highlighting the treatment's ability to create a more even complexion (Figure 3C). When evaluating the reduction of visible borders of melasma patches, 80.6% of responses were rated as Grade 4 or 5, demonstrating a substantial softening of patch edges (Figure 3D). The assessment of overall skin appearance, including texture and luminosity, yielded 79.4% of responses in the top categories, with nearly half rated as Grade 5, indicating a marked enhancement in skin quality (Figure 3E). Finally, the global evaluation of treatment results showed 83.8% of responses in the top two categories, reflecting the experts' high satisfaction with the overall effectiveness of the treatment (Figure 3F). Across all dimensions, the findings demonstrate consistent and significant improvements, providing robust qualitative evidence that medium‐deep chemical peels are a reliable and effective approach for managing melasma.

**FIGURE 3:** Subjective expert evaluation of treatment outcomes following medium‐deep chemical peels for melasma. Blinded expert evaluation of treatment outcomes from eight randomly selected cases. (A) Post‐treatment conditions were correctly identified in 94.4% of cases. (B–F) High ratings (Grade 4 or 5) were observed for pigmentation reduction (87.5%), skin tone uniformity (69.4%), melasma border reduction (80.6%), overall skin appearance (79.4%), and global treatment results (83.8%), confirming the efficacy of medium‐deep chemical peels for melasma management.

### 3.4 Adverse Effects

The most frequently observed adverse effects were hyperpigmentation and erythema. In all cases, prophylactic antiviral therapy with acyclovir at 400 mg administered every 8 h for 15–30 days was employed to prevent herpes simplex infection. One patient exhibited clinical signs and symptoms consistent with herpes, necessitating a switch to valacyclovir at a dosage of 500 mg every 8 h. Although no confirmed cases of infection occurred, oral antibiotic therapy was initiated from the fifth day onward in patients with an initial clinical suspicion and was maintained for 10 days. In most cases, wound healing occurred between 8 and 12 days post‐treatment. One patient experienced an allergic reaction during the healing period.

### 3.5 Representative Clinical Progression

The clinical progression of melasma improvement varied across patients, reflecting differences in baseline pigmentation patterns, anatomical regions treated, and the number of sessions required to achieve visible results. Early and localized improvement was observed following targeted regional applications in most cases. Subsequently, more uniform skin tone and texture were achieved with additional treatments involving broader facial areas. Notably, the degree of improvement often correlated with the timing, extent of anatomical coverage, and the total number of sessions completed. Figure 4 presents four representative cases that exemplify distinct response patterns observed in the study population to illustrate these outcomes more clearly. These examples provide visual context to the objective measurements and qualitative assessments discussed earlier.

**FIGURE 4:** Representative clinical progression of four patients undergoing medium‐depth chemical peel treatment for melasma. Patient 1 (A): shown at the beginning of treatment in March 2023, when the first session was performed on the cheeks. In November 2024, a new session was carried out on the entire cheek area to harmonize the skin tone between previously treated and untreated regions. At follow‐up in January 2025, two months after the last session, notable improvement was observed. Patient 2 (B): shown at baseline in December 2023, when the first phenol peel session was performed on the forehead and nose. In January 2024, the patient developed post‐inflammatory hyperpigmentation (PIH) in the treated areas, which was managed with four microneedling sessions combined with depigmenting agents. In May 2024, a new area—the lateral face—was treated. By June 2024, with PIH regression on the forehead, new hyperpigmented regions had emerged on the lateral face. These were subsequently treated using the same microneedling protocol with lightening agents. A follow‐up image in March 2025 demonstrated significant improvement in both melasma and PIH. Patient 3 (C): shows three stages—at the beginning of treatment in December 2023; one year after initiating treatment; two months after a second session focused on the cheek region (December 2024); and a follow‐up image taken in January 2025, post‐treatment, after three sessions targeting the forehead and cheek. Patient 4 (D): shown at the beginning of treatment in February 2024. The second image, taken in May 2024—three months after the initial phenol peel—shows persistent hyperpigmentation. A second treatment session with trichloroacetic acid (TCA) was performed (not shown in the image sequence). The final follow‐up image was obtained in November 2024, six months after the second photograph and approximately nine months after the initial treatment.

In the first case (Figure 4A), a patient exhibited marked lightening of pigmentation 1 year and 8 months after a treatment initially restricted to the malar region. However, a noticeable difference in skin color persisted between the treated area and the adjacent untreated area. For this reason, a second session was required, which was no longer limited to the malar region but extended across the entire lateral face. Following this broader application, the skin tone became more uniform. The second case (Figure 4B) showed gradual and multi‐stage improvement. The initial treatment in December 2023 involved a phenol peel applied to the forehead and nose. By January 2024, the patient had developed PIH, which had been present for approximately 15 days, suggesting that it emerged shortly after the procedure. The PIH was effectively managed through a total of four monthly microneedling sessions combined with depigmenting agents. In May 2024, the lateral face was treated with a phenol‐croton oil peel with a chemical peel. By June 2024, PIH on the forehead had regressed, but new hyperpigmented areas had appeared on the lateral face. These new lesions were subsequently treated using the same microneedling protocol. At the final follow‐up in March 2025, substantial improvement in both melasma and PIH was observed across all treated regions, reinforcing the importance of personalized, stepwise treatment strategies for patients with evolving pigmentation patterns. The third case (Figure 4C) demonstrated consistent improvement following region‐specific treatments to the cheeks and forehead. Patient 3 is shown at the beginning of treatment in December 2023, when the first session was performed on the cheeks. A second session targeting the same area was completed subsequently. The forehead was also treated in two separate sessions. The image from December 2024 represents a follow‐up conducted 1 year after completing the second treatment session for both regions. A final follow‐up image was taken in April 2025–1 year and 4 months after completing all four treatment sessions (two for the lateral face and two for the forehead)—revealed sustained improvement in pigmentation and overall skin quality. Finally, Patient 4 (Figure 4D) is shown at the beginning of treatment in February 2024. Three months after the initial phenol peel, in May 2024, a partial improvement was observed, with hyperpigmentation still present. A second TCA treatment session was performed (not shown in the image sequence). At the final follow‐up in November 2024–approximately 9 months after the initial treatment—further fading of the hyperpigmentation was evident. This case and the others presented highlight that PIH is a common part of the melasma treatment process with chemical peels. However, when appropriately identified and managed using a tailored protocol, PIH can be effectively controlled, leading to a favorable overall prognosis.

## 4 Discussion

A satisfactory aesthetic appearance has become a significant global concern [21]. Melasma is a chronic hyperpigmentation disorder primarily affecting sun‐exposed areas [2, 22, 23], particularly, the face and is known to impact patients' quality of life (12) significantly. Medium‐to‐deep chemical peels [24], such as TCA [23, 25] and phenol‐croton oil peels, have proven effective treatments for severe or resistant cases of melasma [26]. These treatments work by penetrating more profound layers of the skin, reducing pigmentation, and enhancing overall texture [13, 26]. TCA peels, applied in concentrations ranging from 10% to 65%, consistently deliver reliable results but must be used cautiously in darker skin types to avoid post‐PIH [23, 25]. With their profound dermal remodeling capabilities, Phenol‐croton oil peels are particularly effective for advanced cases [13, 26]. However, they require precise administration to mitigate risks such as systemic absorption and extended recovery times [27]. When these peels are customized to the patient's skin type and paired with appropriate post‐care, they offer transformative outcomes, addressing pigmentation and skin quality [14].

The current study presents a case series involving patients with diverse skin types, reflecting the genetic diversity [28] in a country characterized by significant miscegenation [29]. This diversity posed unique challenges in determining individual phototypes with clinical relevance [29], necessitating a case series design to enable a nuanced and tailored evaluation of treatment efficacy. A key difficulty in melasma studies lies in reliably measuring lesion changes over time while minimizing the influence of external factors. While commonly used, traditional methods like the MASI and colorimetry have notable limitations [20, 30]. MASI's subjectivity and interobserver variability reduce its reproducibility, and it struggles to capture subtle pigmentation changes and improvements in skin texture [31]. Although colorimetry offers more objectivity, it primarily measures skin color changes and may fail to reflect broader clinical and aesthetic effects [32]. The current study addressed these limitations by integrating advanced objective and subjective evaluation methods. The WSI ratio, an enhanced form of colorimetry, provided precise and reproducible measurements of pigmentation changes over time. By analyzing controlled areas, WSI allowed consistent comparisons across different time points. Expert subjective assessments captured qualitative improvements in skin attributes such as texture, luminosity, and overall appearance, complementing this quantitative analysis. The WSI analysis revealed significant improvements in treated areas, with 38 of 42 cases showing positive changes in skin tone. Heatmaps further illustrated uniform reductions in pigmentation, particularly in areas with higher baseline melasma intensity. Subjective evaluations aligned with these findings, with experts correctly identifying post‐treatment images in 94.4% of cases and overwhelmingly rating improvements in pigmentation, skin tone uniformity, and overall skin appearance as Grade 4 or 5.

These findings are consistent with previously published studies demonstrating the efficacy of medium‐to‐deep chemical peels for melasma treatment. The role of chemical peels such as TCA and phenol‐croton oil was revealed to be effective as second‐line therapies for refractory melasma [14]. Similarly, the long‐term effectiveness of phenol‐croton oil peels with varying concentrations of *Croton tiglium* oil was demonstrated, supporting the improvements observed in our study [13]. Moreover, recent evidence reported significant pigmentation reductions following TCA peels, which align with the skin tone and pigmentation improvements documented in our case series [23, 25]. Our findings, combining segmented application and advanced image analysis, reinforce the evidence that medium‐to‐deep chemical peels are a reliable and effective approach for melasma management, particularly when tailored to individual patient characteristics.

Together, these complementary methodologies created a comprehensive and multidimensional evaluation framework, enhancing the reliability and applicability of the results. This approach provided robust evidence for the efficacy of medium‐deep chemical peels in managing melasma, addressing both measurable clinical outcomes and broader aesthetic improvements. This approach provided robust evidence of the effectiveness of medium‐deep chemical peels in managing melasma, addressing both measurable clinical outcomes and broader aesthetic enhancements. By combining objective precision with subjective clinical assessments, this study highlights the effectiveness of TCA and phenol‐croton oil peels in treating diverse patient populations. As a limitation, the study was conducted in a single reference center for quality control. The findings reinforce the importance of personalized treatment strategies for achieving optimal therapeutic outcomes.

In conclusion, medium‐to‐deep chemical peels with phenol‐croton oil or TCA demonstrated significant efficacy in reducing pigmentation, promoting skin regeneration, and enhancing overall skin quality. Quantitative metrics, supported by specialized clinical assessments, validate their role as a targeted and effective approach for melasma management. These results reinforce the potential of the medium‐to‐deep peels as a personalized and evidence‐based therapeutic option for refractory melasma.

## Author Contributions

Study concepts: M.T.S., N.S., M.F.I., W.B.J., I.M.C.C., A.L.O.C., A.L.S.G. Study design: M.T.S., A.L.O.C., A.L.S.G. Data acquisition: N.S., M.F.I., W.B.J., A.L.O.C. Quality control of data and algorithms: M.T.S., A.L.S.G. Data analysis and interpretation: W.B.J., I.M.C.C., A.L.O.C. Statistical analysis: W.B.J., A.L.O.C., A.L.S.G. Manuscript editing: N.S., M.F.I., W.B.J., I.M.C.C., A.L.O.C. Manuscript review: M.T.S., N.S., M.F.I., W.B.J., I.M.C.C., A.L.O.C., A.L.S.G. All authors have read and approved the final manuscript.

## Conflicts of Interest

The authors declare no conflicts of interest.

## Supporting information


**Data S1:** Supporting Information.

**Data S2:** Supporting Information.

## Data Availability

The data that support the findings of this study are available on request from the corresponding author. The data are not publicly available due to privacy or ethical restrictions.

## References

[1] T. J. Lieu and A. G. Pandya , “Melasma Quality of Life Measures,” Dermatologic Clinics 30, no. 2 (2012): 269–280.22284141 10.1016/j.det.2011.11.009

[2] O. Artzi , T. Horovitz , E. Bar‐Ilan , et al., “The Pathogenesis of Melasma and Implications for Treatment,” Journal of Cosmetic Dermatology 20, no. 11 (2021): 3432–3445.34411403 10.1111/jocd.14382

[3] J. McKesey , A. Tovar‐Garza , and A. G. Pandya , “Melasma Treatment: An Evidence‐Based Review,” American Journal of Clinical Dermatology 21, no. 2 (2020): 173–225.31802394 10.1007/s40257-019-00488-w

[4] L. D. Miot , H. A. Miot , M. G. Silva , and M. E. Marques , “Physiopathology of Melasma,” Anais Brasileiros de Dermatologia 84, no. 6 (2009): 623–635.20191174 10.1590/s0365-05962009000600008

[5] B. Torres‐Alvarez , I. G. Mesa‐Garza , J. P. Castanedo‐Cazares , et al., “Histochemical and Immunohistochemical Study in Melasma: Evidence of Damage in the Basal Membrane,” American Journal of Dermatopathology 33, no. 3 (2011): 291–295.21317614 10.1097/DAD.0b013e3181ef2d45

[6] W. Liu , Q. Chen , and Y. Xia , “New Mechanistic Insights of Melasma,” Clinical, Cosmetic and Investigational Dermatology 16 (2023): 429–442.36817641 10.2147/CCID.S396272PMC9936885

[7] A. C. C. Esposito , G. Brianezi , N. P. de Souza , D. C. Santos , L. D. B. Miot , and H. A. Miot , “Ultrastructural Characterization of Damage in the Basement Membrane of Facial Melasma,” Archives of Dermatological Research 312, no. 3 (2020): 223–227.31531731 10.1007/s00403-019-01979-w

[8] S. Rajanala , M. B. C. Maymone , and N. A. Vashi , “Melasma Pathogenesis: A Review of the Latest Research, Pathological Findings, and Investigational Therapies,” Dermatology Online Journal 25, no. 10 (2019): 1–6.31735001

[9] H. Y. Kang , J. S. Hwang , J. Y. Lee , et al., “The Dermal Stem Cell Factor and c‐Kit Are Overexpressed in Melasma,” British Journal of Dermatology 154, no. 6 (2006): 1094–1099.16704639 10.1111/j.1365-2133.2006.07179.x

[10] S. H. Kwon , J. I. Na , J. Y. Choi , and K. C. Park , “Melasma: Updates and Perspectives,” Experimental Dermatology 28, no. 6 (2019): 704–708.30422338 10.1111/exd.13844

[11] H. Y. Kang , I. Suzuki , D. J. Lee , et al., “Transcriptional Profiling Shows Altered Expression of Wnt Pathway‐ and Lipid Metabolism‐Related Genes as Well as Melanogenesis‐Related Genes in Melasma,” Journal of Investigative Dermatology 131, no. 8 (2011): 1692–1700.21562572 10.1038/jid.2011.109

[12] S. H. Kwon , Y. J. Hwang , S. K. Lee , and K. C. Park , “Heterogeneous Pathology of Melasma and Its Clinical Implications,” International Journal of Molecular Sciences 17, no. 6 (2016): 824.27240341 10.3390/ijms17060824PMC4926358

[13] M. B. C. Maymone , F. N. Mirza , D. Steiner , et al., “Comparative Long‐Term Efficacy of Phenol‐Croton Oil Chemical Peels for Persistent Melasma at Varied *Croton tiglium* Oil Concentrations,” Journal of the American Academy of Dermatology 91, no. 2 (2024): 336–338.38574769 10.1016/j.jaad.2024.03.034

[14] R. Sarkar and S. Katoch , “Chemical Peels in Treatment of Melasma,” Dermatologic Clinics 42, no. 1 (2024): 21–32.37977681 10.1016/j.det.2023.06.003

[15] R. A. Agha , C. Sohrabi , G. Mathew , et al., “The PROCESS 2020 Guideline: Updating Consensus Preferred Reporting of CasESeries in Surgery (PROCESS) Guidelines,” International Journal of Surgery 84 (2020): 231–235.33189880 10.1016/j.ijsu.2020.11.005

[16] W. Hu , T. Peng , Y. Huang , et al., “Hyaluronidase‐Powered Microneedles for Significantly Enhanced Transdermal Delivery Efficiency,” Journal of Controlled Release 353 (2023): 380–390.36464062 10.1016/j.jconrel.2022.11.046

[17] J. Schindelin , I. Arganda‐Carreras , E. Frise , et al., “Fiji: An Open‐Source Platform for Biological‐Image Analysis,” Nature Methods 9, no. 7 (2012): 676–682.22743772 10.1038/nmeth.2019PMC3855844

[18] E. S. B. Gomes , L. C. Farias , L. H. Silveira , et al., “Conditioned Fear Stress Increases Bone Resorption in Apical Periodontitislesions in Wistar Male Rats,” Archives of Oral Biology 97 (2019): 35–41.30339914 10.1016/j.archoralbio.2018.10.004

[19] T. A. Guimaraes , L. C. Farias , C. A. Fraga , et al., “Evaluation of the Antineoplastic Activity of Gallic Acid in Oral Squamous Cell Carcinoma Under Hypoxic Conditions,” Anti‐Cancer Drugs 27, no. 5 (2016): 407–416.26849170 10.1097/CAD.0000000000000342

[20] A. G. Pandya , L. S. Hynan , R. Bhore , et al., “Reliability Assessment and Validation of the Melasma Area and Severity Index (MASI) and a New Modified MASI Scoring Method,” Journal of the American Academy of Dermatology 64, no. 1 (2011): 78–83, e71‐72.20398960 10.1016/j.jaad.2009.10.051

[21] N. Scardua , D. P. Rovaris , K. M. S. Moreira , A. L. S. Guimaraes , and M. T. Scardua , “Supraperiosteal Technique Protocol for Forehead Filling With a Mixture of Calcium Hydroxyapatite and Hyaluronic Acid: Double‐Blind, Randomized Controlled Clinical Trial,” Journal of Cosmetic Dermatology 23, no. 12 (2024): 4116–4122.39099032 10.1111/jocd.16488PMC11626347

[22] P. Ghasemiyeh , R. Fazlinejad , M. R. Kiafar , S. Rasekh , M. Mokhtarzadegan , and S. Mohammadi‐Samani , “Different Therapeutic Approaches in Melasma: Advances and Limitations,” Frontiers in Pharmacology 15 (2024): 1337282.38628650 10.3389/fphar.2024.1337282PMC11019021

[23] M. A. Atwa , A. H. Ahmed , H. A. Nada , S. M. Refaey , M. Jafferany , and M. L. Elsaie , “Combined Chemical Peels Versus Trichloroacetic Acid (TCA) for Treating Melasma: A Split Face Study,” Journal of Dermatological Treatment 33, no. 2 (2022): 959–964.32649234 10.1080/09546634.2020.1793888

[24] J. Ocampo‐Candiani , R. Alas‐Carbajal , J. F. Bonifaz‐Araujo , et al., “Latin American Consensus on the Treatment of Melasma,” International Journal of Dermatology 64 (2024): 499–512.39415312 10.1111/ijd.17522PMC11840225

[25] D. Lorenzo‐Rios , G. Arias Berrios , G. I. Cruz Goytia , S. L. Rocafort , and C. N. Brau Javier , “Safety and Efficacy of Trichloroacetic Acid Peels in the Treatment of Melasma: A Split‐Face, Randomized, Prospective Trial in Latin American Women,” Journal of Clinical and Aesthetic Dermatology 17, no. 9 (2024): 28–32.PMC1138697239263263

[26] T. Piamphongsant , “Phenol‐Castor Oil: Modified Peel for Dermal Melasma,” Dermatologic Surgery 32, no. 5 (2006): 611–617.16706754 10.1111/j.1524-4725.2006.32131.x

[27] C. G. Wambier , K. C. Lee , S. L. Soon , et al., “Advanced Chemical Peels: Phenol‐Croton Oil Peel,” Journal of the American Academy of Dermatology 81, no. 2 (2019): 327–336.30550827 10.1016/j.jaad.2018.11.060

[28] S. D. J. Pena , F. R. Santos , and E. Tarazona‐Santos , “Genetic Admixture in Brazil,” American Journal of Medical Genetics. Part C, Seminars in Medical Genetics 184, no. 4 (2020): 928–938.33205899 10.1002/ajmg.c.31853

[29] F. C. Parra , R. C. Amado , J. R. Lambertucci , J. Rocha , C. M. Antunes , and S. D. Pena , “Color and Genomic Ancestry in Brazilians,” Proceedings of the National Academy of Sciences of the United States of America 100, no. 1 (2003): 177–182.12509516 10.1073/pnas.0126614100PMC140919

[30] E. Y. Tay , E. Y. Gan , V. W. D. Tan , et al., “Pilot Study of an Automated Method to Determine Melasma Area and Severity Index,” British Journal of Dermatology 172, no. 6 (2015): 1535–1540.25641313 10.1111/bjd.13699

[31] I. Majid , I. Haq , S. Imran , A. Keen , K. Aziz , and T. Arif , “Proposing Melasma Severity Index: A New, More Practical, Office‐Based Scoring System for Assessing the Severity of Melasma,” Indian Journal of Dermatology 61, no. 1 (2016): 39–44.26955093 10.4103/0019-5154.174024PMC4763693

[32] B. C. K. Ly , E. B. Dyer , J. L. Feig , A. L. Chien , and S. Del Bino , “Research Techniques Made Simple: Cutaneous Colorimetry: A Reliable Technique for Objective Skin Color Measurement,” Journal of Investigative Dermatology 140, no. 1 (2020): 3–12, e11.31864431 10.1016/j.jid.2019.11.003

